# Variation of the Penetration Effort in an Artificial Tissue by Hypodermic Needles

**DOI:** 10.1155/2020/8822686

**Published:** 2020-09-14

**Authors:** Aparecido Carlos Gonçalves, Sidnei Cavassana, Fábio R. Chavarette, Roberto Outa, Samuel J. Casarin, Adalberto Vieira Corazza

**Affiliations:** ^1^Department of Mechanical Engineering (DEM), FEIS, University of State of Sao Paulo (UNESP), Ilha Solteira, SP, Brazil; ^2^Department of Mechanical Engineering, (DEM), FEIS, UNESP, Ilha Solteira, SP, Brazil; ^3^Department of Mathematics, (MAT), FEIS, UNESP, Ilha Solteira, SP, Brazil; ^4^Department of Biofuels, Araçatuba Technology College, FATEC, Sorocaba, SP, Brazil; ^5^Department of Mechanical Engineering, (DEM), FEB, UNESP, Bauru, SP, Brazil; ^6^Faculty of Medicine, Campus of Três Lagoas (CPTL), Federal University of Mato Grosso do Sul (UFMS), Campo Grande, MS, Brazil

## Abstract

Fear of injection-related pain is a drawback to injectable therapy. Hypodermic injections are a cause for great anxiety and reduced adherence to the subcutaneous application of insulin for glycemic control in diabetics or in the treatment of multiple sclerosis, increasing the risk of complications and mortality. Injured or sick people have to undergo several daily injections, forcing them to rotate the veins and regions used to recover from the trauma caused by the perforation of the skin, tissue, muscles, veins, and arteries. People who suffer from type 1 diabetes mellitus (DM1) need to have their glycemic control 3 to 5 times a day and to take insulin up to 3 times a day. In both cases, the patient needs to perforate the skin. To quantify the pain perceived by the patients depends on the evaluation of each patient and therefore is subjective. This study aims to understand the application and self-application of hypodermic injections and decrease pain during its application and the phobia of the patient, following the reasoning that the lower the effort to penetrate the needle, the less trauma in the tissue and therefore the pain provoked. For that, it was analyzed how some of the characteristics of the needle can influence the sensation of pain in the injection. The needle penetration effort was measured in an artificial tissue (substitute skin model) for different cannula diameters, roughness, depth of penetration, lubrication, and angles of the perforating tip bevel. This study aimed to find alternatives to facilitate the application and self-application of hypodermic injections, increase safety and comfort, and reduce the pain intensity perceived by the patient. To do this, the bevel of needles used repeatedly was analyzed in the profile projector and SEM to verify the loss of the profile or the formation of burrs that could hamper the penetration or traumatize the tissue during the reuse of needles. It has also been mechanically analyzed, which can be done to prevent that the needles used in the subcutaneous application do not inadvertently reach the muscle. The greater penetration effort observed in the needles with greater angle of the bevel is responsible for the patient's perception of pain.

## 1. Introduction

Injured or sick people have to undergo several daily injections, forcing them to rotate the veins and regions used to recover from the trauma caused by the perforation of the skin, tissue, muscles, veins, and arteries. People who suffer from Type 1 Diabetes Mellitus (DM1) need to have their glycemic control 3 to 5 times a day and to take insulin up to 3 times a day. In both cases, the patient needs to pierce the skin. The glycemic control is usually done by drilling the fingertips to obtain a small sample of blood for analysis in a portable device and checking the concentration of glucose in the blood. When the level is above normal, insulin is required. If the glycemic index is too low (hypoglycemia), he will need to feed himself, preferably a food rich in carbohydrates. It is a disease that impairs glucose metabolism, which, even at high levels in the bloodstream, is not absorbed by cells. DM1 usually arises due to the destruction of beta cells in the pancreas, responsible for insulin production. This destruction occurs by cellular autoimmune responses, where the body itself destroys its cells, leading to an increase in blood glucose due to nonproduction of insulin. This process worsens to the point that the patient needs to take complementary doses of insulin several times a day. Insulin is a necessary hormone so that the glucose present in the blood stream can be absorbed by the cells and used by our body, providing energy necessary for life. Glucose is the “fuel” that the body's cells use to obtain energy. Without insulin, glucose remains in the bloodstream in increasingly high concentrations and can cause a number of health problems. Insulin cannot be taken orally because it ends up being digested in the stomach, and the bloodstream does not reach where it would be needed. By medical recommendation, insulin should be injected into the subcutaneous tissue, a layer of fat that is just below the skin. There is some research on alternative ways to administer insulin, such as ointments, inhalation, or capsules that dissolve only in the intestine. However, these methods still do not allow the absorption of insulin with the necessary precision for the perfect control of blood glucose.

Many people are afraid to take injection, especially children. This study aims to facilitate the application and self-application of hypodermic injections and decrease pain during its application and the phobia of the patient, following the reasoning that the lower the effort to penetrate the needle, the less trauma in the tissue and therefore the pain provoked.

Different characteristics of the needles were analyzed, such as bevel geometries (needle tip), roughness and cannula diameters, and the effect of lubrication on the needle penetration effort.

To quantify the pain perceived by the patients depends on the evaluation of each patient and therefore is subjective. Even using “pain scales” such as the Visual Analog Scale (VAS), where a linear scale is used to assess pain, covering a range of numbers (0–10 or 0–100), such that the smallest number (0) is indicative of absence of pain and the highest number (10 or 100) is indicative of the worst possible pain. There is also the Gracely Box Scale that incorporates words corresponding to the numbers to detect minor differences in the lower region of the pain scale, such as “painless,” “weak,” “very weak,” and “mild” [1]. The smaller the diameter of the needles and the insertion force, the lower the frequency of painful injections reported by the patients [2].

Among the objectives of this study, the following stand out:

1. To find alternatives to facilitate the application and self-application of hypodermic injections, in the administration of drugs, giving more safety and comfort to the action, aiming at reducing the pain intensity felt by the patient
2. Measure the penetration of needles into an artificial tissue (skin substitute model) by varying the diameters, depth, cannula roughness, lubrication, and bevel angle of the piercing tip
3. Analyze in the profile projector and in the SEM the bevel of needles used repeatedly to verify the loss of the profile or the formation of burrs that can traumatize the fabric during the reuse of needles
4. Mechanically analyze what can be done to prevent that the needles used in the subcutaneous application do not inadvertently reach the muscle

## 2. Theoretical Framework

*Hypodermic Needle and Its Etymology*. “Hypo” has sense of low, under, reduction, and inferior. It comes from the Greek “*ὑπο*” (hupo) and dermal that is related to the skin; hypodermic needle is a tool used to pierce the skin and thus access the interior of living beings, reaching cells, muscles, veins, and arteries.

It is made from a thin metallic strip of austenitic stainless steel. It is then welded and drawn in various lengths and diameters [3]. It is assumed that they were inspired by the animal world where we see stingers and tusks of poisonous snakes that come very close to modern needles (Figure 1).

The dimensions of the hypodermic needle vary according to the purpose of its use and are generally used to inject or to suction fluids, usually coupled to syringes. The diameter (gauge) of the chosen tube usually varies with the viscosity of the fluid and the stress that will be exerted at work. The length is specified according to the distance you want to reach. This tube is called a cannula.

At one end, there is a chamfer called a bevel. This is the tip of the needle and is designed to facilitate tissue perforation. At the other end of the cannula is the cannon. It is generally made of polypropylene or aluminum alloys and has the function of attaching the cannula to the syringe and not allowing leaks. This cannon is manufactured in different colors for easy identification of size. It cannot contain burrs or defects as described in [3]. It must have a conicity of 6% inside to facilitate the placement and removal of the cannon in the syringe. The most usual forms of use are intravenous, subcutaneous, and intramuscular.

Charles Gabriel Pravaz and Alexander Wood were the first to develop a syringe with a hollow needle and thin enough to pierce the skin in 1853. Credits for the evolution of the syringe with the needle are generally attributed to Doctor Alexander Wood (1817–1884) who was born in Scotland. At about the same time, Charles Gabriel Pravaz of Lyon was making a similar syringe that quickly came into use in many surgeries under the name of “The Pravaz Syringe.” Another English doctor, Dr. Francis Rynd, born in Dublin in 1801, worked at Meath Hospital in Dublin. In May 1844, he developed a needle for the introduction of drugs into the vein by dripping. At that time, it was considered possible to administer drugs only orally. In 1845 (eight years before Alexander Wood), Dr. Rynd published an article in the “Dublin Medical Press” reporting how he had successfully used a hypodermic syringe to inject drugs into a patient [4].

There are numerous studies on variables that affect patients' perception of pain during the use of hypodermic needles. According to Norman and Prausnitz [5], studies with diabetics revealed that nearly half of the patients said they would more accurately follow injectable insulin therapy if they knew how to relieve the pain and discomfort in the application. One-third of these patients said they feared their daily injections.

Becton, Dickinson and Company developed a 5-bead needle (Figure 2(b)) which is sharper, smaller in diameter and requires 23% less force for insertion into the skin compared to a traditional 3-bead needle (Figure 2(a)). However, in blind comparison, the 5-bead needle showed no significant difference in pain, preference, ease of insertion, or comfort compared to 3-bead needles. This is consistent with an earlier blind study showing no significant reduction of pain with 5-bead needles as compared to conventional 3-bead needles.

In another study, 29G (disposable Unifine needle for diabetic pen) and 5-bead needles were evaluated as being less painful than 27G and 3-bead needles. However, the fact that 5-bead needles have a smaller diameter and length may confound the possible role of the bevel in the perception of pain. Taken together, these studies suggest that the reduction of insertion force, which has been shown to be statistically significant for 5-bead needles as compared to 3-bead needles cannot be easily perceived by patients as a reduction of pain. In addition, deeper insertion of the needle into the subcutaneous tissue may be equally painful and void the perception of the lower insertion force, which is governed primarily by forces applied to the surface of the skin. Pain becomes subjective because it involves the patient's life history.

According to [6], there are approximately 387 million people with diabetes mellitus in the world, and it is estimated that more than 100 million insulin injections are performed daily. This shows the importance of developing safe, painless, and comfortable needles. Needle makers have sought to develop needles that cause less pain and trauma to the skin, primarily by decreasing the length and diameter of the needle.

However, it is a challenge to maintain an inner lumen large enough so that the force used in the injection application is low and acceptable. This induces a reduction in the wall thickness of the needle limited by the maintenance of its robustness.

A fragile needle would increase the risk of damage to the needle tip during, for example, removal or manipulation of the cap. Needle performance is usually measured by the patients' perception of the pain of the test in a clinical trial or by mechanical tests with measurement of the penetration force through a skin substitute made of polyurethane rubber.

Studies have shown that the penetration force on the skin and on polyurethane rubber is linearly related and that needle insertion without silicone lubrication has increased penetration force and bleeding after withdrawal of the needle, compared to a fully lubricated new needle. However, the lack of silicone did not influence the intensity of the pain. Needles with hooks at the tip caused a greater spike in penetration force than that caused by an intact needle. This is probably due to the lack of the sharp tip and a larger area of contact on the surface when piercing the skin. The increased bleeding was also higher for both, but only needles with hooks larger than 150 *μ*m caused greater pain than a new needle. Therefore, lack of silicone and minor tip damage can cause increased friction when inserting and removing the needle, but this will not necessarily cause more pain.

Confirming previous studies, Clement et al. [7] also came to the conclusion that people perceive the standard process of puncture with needle as painful. This pain is a key factor leading to noncompliance in the treatment of diabetes and other diseases that require puncture with needles. His research aims to reduce the discomfort of needle insertion. It has shown that needle insertion pain varies inversely with the insertion force required to penetrate the skin. Needle designs with smaller diameter, sharper and insertion strategies such as increased insertion velocity reduce the penetration force and deformation associated with tissues and appear to reduce pain and discomfort. In this work, the effect of needle vibration during insertion was studied. It was observed that they led to reductions in puncturing and friction forces.

According to the authors [8, 9] cited by [10], the effect of speed on needle insertion in biological materials was studied, and the shear force of the needle was measured in swine and corpses to construct a surgical simulator for epidural needle procedures. They found that the full force profile does not change with the insertion velocity, while the peak force decreases for faster insertions. It was observed that the mean punction force for needle insertion decreases with increasing insertion velocity in liver samples.

According to studies by [2], needles with smaller diameters and lower insertion force have been shown to be effective in reducing painful injections reported by patients, thus increasing adherence to treatments. In contrast, pain reduction should be balanced due to the need for deep injections, drugs with greater volume, and viscosity, which may be more painful.

Sharpening the needle, lubricating the cannula, and anything else that can reduce insertion force and drug pressure are important parameters that can be improved to reduce pain in needle insertion and administration of the drug.

Another study done to reduce needle penetration effort was made by [11] by biomimetism. North American spines have specialized bristle that have become thorns and are used for self-protection against predator attacks. These spines have the tip with a conical profile and have microscopic back-to-back scales that increase in size as they move away from the tip (Figure 3(A and B)). These allow easy penetration and difficult tissue removal. They contribute to adhesion and unexpectedly reduce the force required for tissue penetration (Figure 3(C, D, and E)). This reduction is due to the surface profile that appears to create tension concentration along the spine, where the diameter of the cross section grows rapidly, facilitating tissue cutting. The scales located in the first geometric transition zone have dual functions. They are mainly responsible for reducing the force required for penetration and are also responsible for the greater impact on tissue adhesion strength in the 0–2 mm and 2–4 mm regions (Figure 3 (F and G)).

By decreasing the penetration effort, besides reducing pain during needle insertion, we reduce the risks of buckling and needle breaking during biomedical applications, such as anesthesia, abscess drainage, and the development of tissue adhesives mechanically interconnected.

The needle shall be made with a cannula in accordance with [12], which prescribes the material used for its manufacture as austenitic stainless steel of one of the types given in Table 1.

The Unified Numbering System (UNS) is managed by the American Society for Testing & Materials (ASTM International) and Society of Automotive Engineers (SAE International). The UNS number per se does not constitute a complete specification of the material because it does not lay down any requirements for its properties, heat treatment, form, or quality. American Iron and Steel Institute (AISI) defends the interests of the North American Steel Industry and normalizes its products.

## 3. Materials and Methods

This research is characterized as experimental, quantitative, and comparative. Here, we describe the main equipment and methodologies used throughout its development.

The cannulas were manufactured using 304L stainless steel microtubes provided in the external diameters of 0.6 mm–0.8 mm–1.0 mm–1.2 mm–1.4 mm and 500 mm length (see Figure 4).

The tubes were sanded with 3 M water slurries in the measurements (JIS) P120, P180, 400, 600, and 1200.

A Dremel (Mini Mite) manual grinding model 750–10,000 rpm was also used.

The cannulas were cut with Ø 22.2 mm × 0.6 mm (Ø 7/8″ × 0.023″) cutting discs—Aluminum Oxide for Chrome Cobalt (Dentorium Products Co., Inc., USA).

For the polishing of the bevel, fabric discs with Ø 25 mm were used. Nylon brushes were used to remove burrs from the bevel. A 1/8″-3/32″-1/16″-1/32″ Tweezers Kit was used for grinding and roughening the cannula. A mini bench vise with 1″ was also used.

The bevel manufacturing template was made of aluminum (Figure 5), designed to aid in the cutting and polishing of the bevel. It contains grooves for fixing the cannulas to be machined at angles of 15°, 30°, 45°, 60°, 75°, and 90° with respect to the horizontal axis.

Figure 6 illustrates the design made for the manufacture of the bevel template.

Each cannula was positioned in the template at the angles marked on the inside. The sharpening of the cannula tips was done by manual sanding, using a flat surface as the base and the template as an angle reference. On them were placed the sanding for the initial thinning until finishing, following the order: (JIS) P120, P180, 400, 600, and 1200.

After sanding, the bevel was brushed lightly with the nylon brush to eliminate burrs and after brushing, the bevel was polished with fabric disc. After polishing, the cannula and the bevel were cleaned with alcohol and compressed air.

The Mecmesin Digital Dynamometer (Advanced Force Gauge) was used in conjunction with the base and has an uncertainty level ±0.1% of the total scale) with a capacity of 50 N. The Mecmesin dynamometer (Figure 7) has a MultiTest 2.5-d motorized test base that allows testing of up to 2.5 kN traction and compression.

Emperor Lite software was used to obtain and process data collected from the dynamometer. It is possible to interpret the results through graphs that can be viewed individually or superimposed to facilitate comparisons and production of test reports.

Human skin was simulated by a modeling described below. The model (Figure 8) was made of siliconized plastic resin (polyurethane). Gelatinous material contains 3 layers that simulate the skin, subcutaneous tissue, and a layer of muscle. It is usually used by medical, pharmacy, or nursing students for suture training and intradermal, hypodermic, and intramuscular injection. The layers are approximately 3 mm (cutaneous); 9 mm (subcutaneous); and 15 mm (muscular).

The dynamometer was installed in the motorized test base to start the tests. To fix the needles, a tweezers was placed in the device (Figure 9) that allowed the positioning of the needles by the tightening of a butterfly.

The base was adjusted for forward and backward speed of 100 mm/min (insertion and withdrawal of the needle in the simulator model of the human skin).

The test needle in the dynamometer clamp was positioned vertically using the motorized base rod as a reference, at a distance of approximately 3 mm from the model, to begin recording the needle penetration and withdrawal efforts in the human skin simulator model.

The zero was set on the needle shift gauge. He advanced the needle at the programmed speed (100 mm/min) until reaching a depth of approximately 20 mm in the simulator model of the human skin. Shortly after reaching the depth of 20 mm, the needle was withdrawn at the programmed speed (100 mm/min) until the tip (bevel) came out completely from the simulator model of the human skin.

Records have been saved using the Emperor Lite Software. The registers of the forces involved in the test were saved in the computer for later analysis and interpretation of the results of the variations in the angle of the bevel, the diameter of the cannula, its roughness, and the influence of the lubrication. The lubrication was done by passing a cotton swab dipped in silicone oil (polydimethylsiloxane) on the surface of the cannula and cleaned with absorbent paper. Tests were performed with the cannula with Ø 0.6 mm–Ø 0.8 mm–Ø1.0 mm–Ø1.2 mm–Ø1.4  mm with level angles of 15°, 30°, 45°, 60°, 75°, and 90°. Tests were performed with cannulas with Ø 0.6 mm, with bevel angles of 15°, with roughness of the cannula altered by sanding with P120 and P180.

## 4. Results

Comparative analyses were performed to understand the influence of some variables on the penetration effort in artificial tissue, such as diameter of the cannula, angle at the tip of the needle (bevel), roughness of the cannula, direction in the roughness grooves, and depth of penetration. Practical tests were also made through the reuse of hypodermic needles. The needle was inserted into the artificial tissue to observe the depth reached.

In the studies on the influence of the variation of the bevel angles (15°, 30°, 45°, 60°, 75°, and 90°), the diameters of the cannulas were fixed.  Figure 10 presents the results obtained.

Figure 10 shows the temporal course of the force of 6 bevel angles: (a) for the cannula with 0.60 mm in diameter, (b) for the cannula with 0.80 mm in diameter, (c) for the cannula with 1.00 mm in diameter, (d) for the cannula with 1.20 mm in diameter, and (e) for the cannula with 1.40 mm in diameter. Looking at Figure 10, it is observed that

- with 0.60 mm in the diameter of the cannulas, the force reaches the maximum for bevel angle of 60°, with a magnitude of 1.6 N
- with 0.80 mm in the diameter of the cannulas, the force reaches the maximum for bevel angle of 75°, with a magnitude of 1.75 N
- with 1.00 mm in the diameter of the cannulas, the force reaches the maximum for bevel angle of 90°, with a magnitude of 1.75 N
- with 1.20 mm in the diameter of the cannulas, the force reaches the maximum for bevel angle of 90°, with a magnitude of 2.6 N
- with 1.40 mm in the diameter of the cannulas, the force reaches the maximum for bevel angle of 90°, with a magnitude of 3.0 N

Figure 10 represents the force applied against the time of its application, and the duration between penetration and removal of the needle lasted 25 seconds for all cases. The maximum forces occurred between 7.5 and 12.5 seconds. The force of withdrawal of the needles, as observed in the figure, was lower than the insertion force for all diameters of the cannulas.

The studies on the influence of needle diameter variation (Ø 0.6 mm, Ø 0.8 mm, Ø 1.0 mm, Ø 1.2 mm, Ø 1.4 mm) on the penetration effort of the cannulas, maintaining fixed angle of the bevel.  Figure 11 presents the results.

Keeping the bevel angles constant and varying the cannula diameters, the greatest forces are observed for the largest diameters. The needle with a diameter of 6 mm and bevel angle of 15° showed the lowest application force (1 N), according to Figure 11(a).

The needle with a diameter of 1.4 mm and bevel angle of 90° showed the highest application force (3 N) as shown in Figure 11(f).

The studies on the influence of needle lubrication with Ø 0.6 mm cannulas, made with silicone oil, on the penetration force in artificial fabric, sanded in the longitudinal direction of the insertion, with P180 and P120 sandpaper result in the following behaviors, indicated in Figure 12.

Figure 12 shows the effect of lubrication on the application force. Needles sanded and applied without lubricants showed greater application strength (blue color) compared to sanded and polished when lubricated.

In the studies on the influence of the angle of the bevel of needles with cannulas of Ø 0.6 mm to Ø 1.4 mm, in the force for initial puncture of the artificial skin, we obtained the following results, expressed in Figure 13.

Figure 13 shows that as the bevel angle is increased to the same diameter, the force of the application increases. The same figure also shows that for the same bevel angle, the application force increases as the diameter increases. The best option, in the case studied, was the needle with 6 mm in diameter and bevel angle of 15. The worst option was the needle with 1.4 mm in diameter with bevel angle of 90.

In the studies on the influence of needle diameters on the strength for initial puncture of the artificial skin, for bevels of 15°, 30°, 45°, 60°, 75°, and 90°, the following results, expressed in Figure 14, were obtained.

Figure 14 shows that the larger the needle diameter, the greater the force applied to puncture (pierce) the skin during penetration. It is also observed that the greater the bevel angle, keeping a diameter fixed, the greater this force will also be. The lowest force was 0.25 N for the 6 mm diameter needle with a bevel angle of 15° and the highest force was 2.9 N for the 1.4 mm diameter needle with a bevel angle of 90°.

### 4.1. Analysis of Results

We analyzed some factors that affect pain reported by patients during subcutaneous administration of medication. Based on Clement at al. [7], the premise of this study is that the lower the penetration force of the hypodermic needle, the lower the perceived pain in the patient.

In agreement with Hirsch et al. [14], we analyzed some factors that influence pain in the application of subcutaneous insulin injection. The factors analyzed were the depth of needle penetration, diameter, polishing, needle tip geometry, and lubrication of the cannulas.

The injected volume and the drug (which may include preservatives and solvents) that according to Hirsch et al. [14] may also affect the perception of pain were not analyzed.

In tests performed by keeping the diameter of the cannula fixed and varying the angle of the bevel, it was concluded that the greater the angle of the bevel, the greater the effort to penetrate the artificial tissue.

In the tests made with the bevel angle fixed and the cannula diameter varied, it was concluded that the larger the cannula diameter, the greater the effort to penetrate the artificial tissue.

In the tests made in cannulas with Ø 0.6 mm on the influence of its roughness, altered by sanding transversal to the direction of insertion, with sandpapers P120 and P180, it was concluded that the effort for penetration in the artificial fabric increased in comparison to the normally polished cannula.

In the tests made in cannulas with Ø 0.6 mm on the influence of its roughness, altered by longitudinal sanding to the direction of insertion, with sandpapers P180, it was concluded that the effort to penetrate the artificial tissue did not change compared to the normally polished cannula. In the tests made with P120 sandpaper, it was concluded that the effort to extract the needle in the artificial tissue was reduced by around 20% compared to the normally polished cannula.

In the tests made on the influence of the sanding direction (transverse and longitudinal to the direction of insertion) on the penetration force in an artificial fabric, made with P180 sanding in cannula with Ø 0.6 mm, there was no significant difference. In the tests made with P120 sandpapers, there was a reduction of approximately 20% in the force measured for extraction of the sanded needle in the longitudinal direction compared to the cross-sanding in the direction of insertion and the polished cannula.

In the tests on the influence of lubrication, with silicone oil on needles with cannulas with Ø 0.6 mm, in the penetration force in artificial fabric sanded in the longitudinal direction to the insertion, with P180 sandpaper, a reduction of approximately 15% in needle penetration force and 50% reduction occurred in force for needle extraction from artificial tissue.

In the tests on the influence of lubrication, with silicone oil on needles with cannulas with Ø 0.6 mm, in the penetration force in artificial fabric sanded in the longitudinal direction to the insertion, with sandpapers P120, also a reduction of approximately 15% occurred in the needle penetration force, but there was no reduction in the force for extraction of the needle from the artificial tissue. However, when compared to needles with polished and also lubricated cannulas, there was no improvement in the penetration force or extraction of the needle.

In the tests on the influence of the angle of the bevel of needles with cannulas of Ø 0.6 mm to Ø 1.4 mm, in the force for initial puncture of the artificial skin, it was possible to conclude that there is an increase in the penetration force with the increase of the bevel angle.

In the tests on the influence of the needle diameters, in the strength for initial puncture of the artificial skin, a bevel of 15°, 30°, 45°, 60°, 75°, and 90° was also observed an increase in the penetration force with the increase of the angle of the bevel.

In the practical tests for the reuse (not recommended) of hypodermic needles used in pens, 31G × 5 mm BD needles, no breakdowns were found that could have been caused by repeated insertions.

The penetration force increases continuously with increasing the depth that the needle reaches the artificial tissue. There are slight variations in strength when the needle passes from one layer to another in the artificial tissue (skin for fat and fat for muscle). The penetration force has a slight reduction soon after the transposition of the layers which is probably due to the increase of the penetration velocity, due to the elastic deformation of the tissue.

## 5. Conclusions

Based on the premise of this study, the lower the penetration force of the hypodermic needle is the patient's perception of pain, it was concluded that the pain felt in the penetration decreases with the reduction of the diameter of the needles and with the angle of the bevel. The limitation of reduction of the cannula diameter and wall would be in the embrittlement of the needle and in the flow rate of the drug. In the practical tests, it is also noticed that an insulin glargine flow rate above 0.04 ml/s or with a cooling temperature (approximately 8°C) causes the patient to complain of pain.

The lubrication of the cannula presented good results reducing the penetration force and the force for extraction of the needle.

The roughness of the cannula increased by longitudinal sanding with P120 sandpaper showed a reduction of approximately 20% in the force measured for extraction of the sanded needle in the longitudinal direction compared to the sanding transverse to the direction of insertion and the polished cannula. The purpose of the sanding was to simulate the scales on the tip of the spines of the North American hedgehog. These scales reduce the penetration force by approximately 50% according to studies by Cho et al. [11].

In the tests where hypodermic needles 31G × 5 mm, used in pens for insulin application, were reused, no failure was found due to repeated insertions. It was observed since before each new application, the needle was analyzed with a magnifying glass to make sure that its tip was in excellent condition. Also, after each insertion of the needle into the artificial skin, an insulin unit was injected “empty” (0.01 ml) in order to verify the nonobstruction of the needle by the anterior insertion.

In the practical tests to evaluate the depth achieved by 31G × 5 mm needles in artificial tissue, it was concluded that the needle can reach the muscle tissue depending on the speed and pressure exerted during the application. This can cause variations in insulin absorption, which may cause hypoglycemia or hyperglycemia to the patient.

## Figures and Tables

**Figure 1:** Hypodermic needle.

**Figure 2:** Needle tips: (a) 3-bevel tip; (b) 5-bevel tip. Source: Norman and Prausnitz [5].

**Figure 3:** SEM photos of the spine and analysis of penetration and removal forces in muscle tissue. Source: Cho et al. [11]. Note: A—North American porcupine thorn. B and C—images showing the microstructure of the tip and tip base, respectively. D—the fluorescence image that allows the visual delineation of the geometry of the scales. E—image showing the microstructure of the tip of the porcupine's spine. F—the representative plots of force versus extension show puncture, penetration, and removal of scaleless, nonscaled spine and African porcupine from tissue (scale bars: 100 *μ*m). The red arrows indicate resistance to tissue removal (not observed in others). G—summary of experimental values obtained from the penetration/removal of the scaly, scaleless, G 18 needle and African porcupine spine. Source: Cho et al. [11].

**Figure 4:** Drawn tubes for the manufacture of cannulas.

**Figure 5:** Bevel manufacturing template.

**Figure 6:** Design of the bevel template.

**Figure 7:** Mecmesin dynamometer set.

**Figure 8:** Simulator model of human skin.

**Figure 9:** Tweezers installation.

**Figure 10:** Graphs on the influence of the variation of the bevel angles (15°, 30°, 45°, 60°, 75°, and 90°), keeping the diameters of the cannulas fixed. (a) Graphic 1—cannula with *φ* 0.60 mm. (b) Graphic 2—cannula with *φ* 0.80 mm. (c) Graphic 3—cannula with *φ* 1.00 mm. (d) Graphic 4—cannula with *φ* 1.20 mm. (e) Graphic 5—cannula with *φ* 1.40 mm.

**Figure 11:** Influence of the variation of the needle in the effort of penetration of the cannula, keeping the angle of the bevel fixed.

**Figure 12:** Influence of lubrication of needles with Ø 0.6 mm cannulas, made with silicone oil, in the force of penetration in artificial fabric, sanded in the longitudinal direction of the insertion, with sandpapers (a) P180 and (b) P120.

**Figure 13:** Influence of the angle of the bevel of needles with cannulas of Ø 0.6 mm to Ø 1.4 mm, in the force for initial puncture of the artificial skin.

**Figure 14:** Influence of the diameters of needles, in the force for initial puncture of the artificial skin, for bevels of 15°, 30°, 45°, 60°, 75°, and 90°.

**Table 1:** Types of stainless steel for tubes.

NBR ISO 9626/2003 [12]	NBR ISO 15510/2014 [13]
X2CrNi18-9	304L (AISI)
X5CrNi18-9	304 (AISI)
X6CrNiNb18-10	347 (AISI)
X5CrNiMo17-12-2	316 (AISI)
X6CrNiMoTi17-12-2	S31635 (UNS)
X6CrNiMoNb17-12	S31640 (UNS)

Source: adapted from [12, 13].

## Data Availability

The data used to support the study can be available upon request to the corresponding author.
